# Assessing the outcomes of prescribing angiotensin converting enzyme inhibitors and angiotensin receptor blockers for COVID-19 patients

**DOI:** 10.1016/j.heliyon.2023.e19373

**Published:** 2023-08-22

**Authors:** Wissam Mekary, Souha Fares, Farah Abdulhai, Gaelle Massoud, Marwan Refaat, Mathias Mericskay, George W. Booz, Fouad A. Zouein

**Affiliations:** a Department of Pharmacology and Toxicology, American University of Beirut Medical Center, Faculty of Medicine, Beirut, Lebanon; b The Cardiovascular Renal And Metabolic Diseases Research Center of Excellence, American University of Beirut Medical Center, Faculty of Medicine, Beirut, Lebanon; c Hariri School of Nursing, Faculty of Medicine, American University of Beirut, Beirut, Lebanon; d Department of Internal Medicine, Cardiovascular Medicine/Cardiac Electrophysiology, American University of Beirut Faculty of Medicine and Medical Center, Beirut, Lebanon; e Clinical Research Institute, American University of Beirut Medical Center, Beirut, Lebanon; f Department of Gynecology and Obstetrics, Division of Reproductive Sciences & Women's Health Research, Johns Hopkins Medicine, Baltimore, USA; g Department of Signaling and Cardiovascular Pathophysiology, UMR-S 1180, Inserm, Université Paris-Saclay, France; h Department of Pharmacology and Toxicology, School of Medicine, University of Mississippi Medical Center, Jackson, MS, USA

**Keywords:** SARS-CoV-2, Renin angiotensin aldosterone system, Cardiac biomarkers, Inflammatory biomarkers, Inflammation, Cytokines

## Abstract

**Background:**

Patients with heart failure were affected severely by COVID-19. Most heart failure patients are on guideline directed medical therapy, which includes ACE inhibitors (ACEI) and ARBs. These medications were controversial at the beginning of the pandemic due to their interplay with the receptor that SARS-CoV-2 binds in the lungs. We investigated the effect that ACEI and ARB had on patients with hypertension, coronary artery disease, and heart failure.

**Methods:**

We recruited 176 patients with COVID-19 infection and cardiovascular comorbidities at the American University of Beirut Medical Center in Lebanon. Of these, 110 patients were taking ACEI or ARB and 66 were not. We collected clinical data and looked at inflammatory markers such as CRP and IL-6 and cardiac markers such as troponin T. We also reported the incidence of ARDS, sepsis, and death of each patient, and compared the 2 groups.

**Results:**

We found that patients taking ACEI and ARB had a statistically significant decrease in levels of troponin T, IL-6, and CRP compared to patients not taking these medications (p < 0.05). We found no difference in rates of ARDS, sepsis, or death between the 2 groups.

**Conclusion:**

Inhibition of the renin-angiotensin-aldosterone-system had no effect on the mortality of patients with COVID-19 and on their overall disease progression. However, it may be beneficial not to stop these medications as they decrease inflammation in the body and the levels of troponin, which are related to increased stress on the heart.

## 1 Introduction

The SARS-CoV-2 outbreak emerged in Wuhan, China in early December 2019 and spread rapidly throughout the world, resulting in an ongoing pandemic (COVID-19) with serious global health burden [1]. The disease manifestation varies from one person to another. The disease may be asymptomatic or mild for many patients [2]. A small proportion of patients, most of them having concomitant pulmonary and cardiovascular disease, suffer from severe to critical disease [3]. COVID-19 may present with respiratory distress requiring additional oxygen therapy or cardiovascular manifestations, such as heart failure exacerbation or myocardial injury [4,5].

Although being a new virus, SARS-CoV-2 belongs to a family of viruses, the coronaviruses which have been studied in previous outbreaks in 2002 and 2012 [5]. Previous studies on the SARS viruses showed that the binding site of these respiratory viruses is angiotensin converting enzyme 2 (ACE2) in alveolar tissues [6]. These ACE2 receptors are part of the renin-angiotensin-aldosterone-system (RAAS), which plays an important role in the regulation of blood pressure and the hemodynamics of the human body [7].

The mechanism of lung damage due to COVID-19 infection is thought to be caused, in part, by downregulation of ACE2 by the body due to the offending virus. The downregulation may lead to toxic accumulation of Ang II – a substrate metabolized by ACE2 – in the lungs and the circulation, inducing lung injury and myocarditis [8,9]. Prescribing drugs that interact with the RAAS could potentially have either a beneficial or detrimental effect on the COVID-19 disease progression. It is conceivable that taking an angiotensin converting enzyme inhibitor (ACE_I_) or an angiotensin receptor blocker (ARB) would lead to an increase in the expression of ACE2 [6]. This would lead to a higher virus burden binding in the lungs and more severe infection [10]. Alternatively, ACE2 plays an important role by converting Ang II into Ang (1–7) which is tissue protective and a vasodilator [10]. The increase in ACE2 caused by taking ACE_I_ and ARB would offset the burden of Ang II, which causes lung and heart injury. Moreover, ACE_I_ and ARB are thought to be cardioprotective and prevent abnormal cardiovascular remodeling by blocking signaling downstream of the angiotensin II type 1 (AT_1_) receptor [11].

Whether ACE_I_ and ARBs are correlated with beneficial or detrimental clinical outcomes remains to be determined. Based on both previous and emerging evidence, we hypothesized that COVID-19 patients on ACE_I_ and ARBs exhibit beneficial cardiovascular clinical outcomes during the symptomatic phase and after recovery.

## 2 Methods

### 2.1 Study design

This study is a retrospective study. The study was approved by the American University of Beirut's Institutional Review Board (IRB). IRB ID: BIO-2020-0362.

### 2.2 Clinical setting and patient recruitment

The American University of Beirut Medical Center (AUBMC) provided medical care for COVID-19 patients in its emergency department (ED), COVID-19 Unit, and COVID-19 Intensive Care Unit (ICU). This study included COVID-19 positive patients at AUBMC who had a medical history of any cardiovascular disease (CVD). The focus was on patients with heart failure or patients predisposed to have heart failure and who have coronary artery disease (CAD) and/or hypertension (HTN). We recruited patients who presented to the ED, and patients who were admitted to the COVID-19 unit and COVID-19 ICU. Three hundred twenty-eight patient records were screened. After excluding patients who were immunosuppressed or had active cancer, and patients who were admitted for two days or less, the final number of patients enrolled in the study was 176, of whom 110 were taking ACEi or ARB and 66 were not.

### 2.3 Data collection

Patients provided informed consent when recruited. Their medical record number (MRN) was used to open their EPIC charts and collect data from their COVID-19 admission. The MRN was replaced by a study code. Data were collected, deidentified, and entered into SPSS for analysis.

### 2.4 Variables

We recorded patient demographic characteristics such as age, weight, gender, date of disease course since the start of symptoms, and their cardiovascular and pulmonary history. Pulmonary history was reported as either the patient had any pulmonary disease (chronic obstructive pulmonary disease, asthma, bronchiectasis, and pulmonary hypertension) or did not have any. Cardiovascular disease history was reported as heart failure or predisposition to heart failure (HTN, CAD). We reported the type of treatment the patients were receiving for their heart failure, CAD or HTN and categorized them into two groups: control group-one included patients not taking an angiotensin converting enzyme inhibitor (ACEI) or angiotensin receptor blocker (ARB); Study group-two included patients taking either an ACEI or ARB.

We outlined the treatments given for the COVID-19 or any suspected bacterial coinfection. At the time of the study, steroids, Remdesivir, Tocilizumab, Ivermectin, and convalescent plasma were used to treat COVID-19. For any suspected bacterial coinfection, a wide variety of antibiotics were used. For outcomes, we focused on inflammatory markers such as C-reactive protein (CRP), pro-calcitonin, and interleukin-6 (IL-6) and the cardiac marker troponin T at the time of admission and during the hospital stay. We reported the vascular marker D-dimer along with the occurrence of deep vein thrombosis (DVT) or pulmonary embolism (PE). We reported the discharge state of the patient as alive or dead.

### 2.5 Ethical considerations

Informed consent was given by the patients to use their medical record for this study. Patient information was confidential and was kept protected by deidentification and storage in a separate file on the primary investigator's computer that is password protected.

### 2.6 Sample size calculation and statistical analysis

#### 2.6.1 Sample size calculation

Sample size calculation was done based on the effect of ACEI/ARBs and controls on the primary outcomes, thus the results of the secondary outcomes were considered as exploratory only. Sample size for linear regression assuming a medium effect size of 0.15, 10 predictors (including ACEI/ARBs vs Controls) and an alpha of 0.05/4 = 0.0125 to account for the multiple inflammation markers considered (thus, multiple linear regression models) a minimum of 160 subjects is needed. Sample size calculation was done using GPower version 3.1.9.7.

#### 2.6.2 Statistical analyses

Continuous variables were summarized by means and standard deviations or medians and inter-quartile ranges as appropriate, while categorical variables were summarized by counts and percentages. Characteristics of patients with missing data were compared to those without missing data to assess the risk of bias. Unadjusted associations between study outcomes and potential predictors were assessed using independent-samples *t*-test, Mann-Whitney *U* test, chi-square test, and the Fisher's exact test as appropriate. Adjusted associations were assessed using linear regression for continuous outcomes and logistic regression for dichotomous outcomes. Due to the non-normality of the continuous variables and the small number of subjects in some categories of the categorical variables, bootstrap estimates and 95% confidence intervals for the linear regression coefficients and the odds ratios were generated and reported. Variables that had a p-value <0.2 at the univariate level were entered in the multivariable models to account for potential confounding. Statistical analyses were performed using SPSS v28.0.1.1(14). All tests were two-tailed and a p-value less than 0.05 was considered significant.

## 3 Results

### 3.1 Background characteristics

A total of 176 patients were included in the study (110 taking ACE_I_ or ARB and 66 that were not). Most of the patients were males (128 patients, 73%) and belonged to the ACEI/ARB group (86 patients, 78%). Female patients were equally divided between the control group and the ACE_I_/ARB group. There was a statistically significant difference between the 2 genders (p = 0.001). There was no statistically significant difference between the 2 groups regarding age, weight, day of symptoms at presentation to the hospital, comorbidities, and COVID-19 treatment (Table 1).

**Table 1:** Comparison in demographic parameters, comorbidities and treatments between the study group and the control group.

Variables	Control (N = 66)	ACEI/ARB (N = 110)	P-value
Demographics N (%) N (%)			
Male	42 (64)	86 (78)	0.001
Female	24 (36)	24 (22)	–
Age (years) (mean ± SD)	69.9 ± 12.7	68.5 ± 11.9	0.378
Weight (kg) (mean ± SD)	82.4 ± 18.8	88.6 ± 17.4	0.344
Day of symptoms on admission (mean ± SD)	7.27 ± 3.64	7.42 ± 3.45	0.61
Comorbidities			
Heart Failure	6 (9)	16 (15)	0.352
Pre-Heart Failure^a^	60 (91)	94 (85)	–
Pulmonary disease	10 (15)	17 (16)	1
No Pulmonary disease	56 (85)	93 (84)	–
COVID-19 treatment			
Steroids	63 (96)	95 (86)	0.112
Remdesivir	38 (58)	56 (51)	0.649
Tocilizumab	25 (38)	38 (35)	0.767
Ivermectin	38 (58)	61 (56)	0.922
Convalescent Plasma	19 (29)	34 (31)	0.916
Bacterial co-infection treatment			
Antibiotics	43 (65)	67 (61)	0.842

a Pre-Heart Failure” designates patients who are pre-disposed to developed heart failure and include patients who had coronary artery disease, hypertension, and arrhythmias (such as atrial fibrillation and atrial flutter).

### 3.2 Unadjusted analysis

The main predictor in this study was whether the patient is or is not taking ACE_I_ or ARB in the setting of CVD. The control group included patients who are not taking ACE_I_ or ARB. In the unadjusted analysis of the main outcomes, we found a significant decrease (p < 0.05) in peak IL-6, peak CRP, peak troponin T within the first 24 h of admission and peak troponin T during the whole hospitalization, in patients taking ACE_I_ and ARB compared to the control group (Table 2). No statistically significant differences between the control and the ACE_I_/ARB group were found for any of the secondary outcomes considered: elevated troponin on admission, ARDS, sepsis and death (Table 3).

**Table 2:** Unadjusted analysis of the main outcomes.

Main Outcomes	ACEi/ARB (mean ± SD) N = 110	Control (mean ± SD) N = 66	CI (95%)	P-value
Peak IL-6 (pg/mL)	148.5 ± 281.92	507 ± 1306.89	(-650.35; −66.68)	<0.001
Peak troponin first 24hrs (ng/mL)	0.0299 ± 0.0605	0.0892 ± 0.4	(-0.14; 0.021)	0.018
Peak troponin (ng/mL)	0.044 ± 0.089	0.146 ± 0.506	(-0.204; 0)	<0.001
Peak CRP (mg/L)	97.47 ± 66.35	128.49 ± 98.01	(-55.62; −6.4)	0.004

**Table 3:** Unadjusted analysis of the secondary outcomes.

Secondary outcomes	ACE/ARB (%) N = 110 (62%)	Control (%) N = 66 (38%)	P-value
ARDS (Yes)	25 (22.7)	12 (18.1)	0.347
Death (Yes)	29 (26.4)	23 (34.8)	0.29
Elevated troponin on admission (Yes)^a^	25 (22.7)	22 (33.3)	0.342
Sepsis (Yes)	20 (18.2)	13 (19.7)	0.902

a For elevated troponin on admission, 10 subjects did not have their troponin measured on admission.

### 3.3 Multivariable linear regression analysis (adjusted) for the main outcomes

Using bootstrap linear regression, we analyzed the relationship between the predictors and the main outcomes. Predictors considered for the multivariable analysis were: day of the disease course on admission (days since symptoms started), gender, age, weight, pulmonary disease history (yes/no), CVD disease ([HTN, CAD] or heart failure). When looking at the peak troponin T on admission (within 24 h of admission), older patients had a higher level of troponin, whereas patients taking ACE_I_ or ARB had lower levels of troponin. If we measure the peak troponin levels within the whole admission, patients taking ACE_I_ or ARB and heavier (higher BMI) patients had lower levels of troponin T. From an inflammatory standpoint, peak IL-6 levels were lower in patients taking ACE_I_ or ARB and patients who presented late after the start of their symptoms. Peak CRP levels were also lower in patients taking ACE_I_ or ARB and who were heavier, whereas patients who presented later in the symptomatic phase had higher CRP levels (Table 4).

**Table 4:** Multivariable linear regression analysis for the main outcomes.

Main Outcomes Model	Predictors	Estimates	P value	Bootstrap CI
**Peak Troponin 1**st **24hrs**	ACEi/ARB	−0.052	0.192	(-0.131; 0.026)
	Age	0.005	0.002	(0.002; 0.008)
**Peak Troponin hospitalization**	ACEi/ARB	−0.084	0.125	(-0.191; 0.023)
	Weight	−0.003	0.044	(-0.006; 0)
**Peak IL-6**	ACEi/ARB	−336	0.025	(-630;-42)
	Day at presentation	−31	0.142	(-73; 10)
**Peak CRP**	ACEi/ARB	−33.27	0.019	(-61;-5.5)
	Day at presentation	4.766	0.013	(1; 8.5)
	Weight	−0.273	0.47	(-1; 0.471)

### 3.4 Multivariable logistic regression analysis for the secondary outcomes

Analysis of the secondary outcomes were not powered a priori and thus were conducted for exploratory purposes. Using bootstrap binary logistic regression, we analyzed the relationship between the predictors and the secondary outcomes: Elevated troponin T on admission (Table 5), ARDS (Table 6), death (Table 7), and sepsis (Table 8). Our data shows that older patients and patients known to have heart failure were more likely to have elevated troponin on admission. Moreover, male patients were at higher risk of developing ARDS. Patients with heart failure were more prone to develop sepsis and die from COVID-19 infection or its complications.

**Table 5:** Multivariate logistic regression analysis for elevated troponin T (>0.007 ng/mL) on admission.

Elevated troponin T on admission - Model	Yes Mean ± SD Or N (%)	No Mean ± SD Or N (%)	OR	Bootstrap CI
ACEi/ARB				
Yes	25 (25.3)	74(74.7)	0.419	(0.168; 1.045)
No	22 (35.5)	40 (64.5)		
Day at presentation	6.28 ± 4.07	7.89 ± 3.31	0.944	(0.835; 1.067)
Age (year)	76.77 ± 9.69	65.23 ± 11.59	1.082**	(1.033; 1.134)
Gender				
Male	30 (25.4)	88 (74.6)	0.837	(0.311; 2.251)
Female	17 (39.5)	26 (60.5)		
Weight (Kg)	80.42 ± 19.89	90.07 ± 17.32	0.987	(0.96; 1.015)
Pulmonary History				
Negative	36 (26.9)	98 (73.1)	0.566	(0.152; 2.1)
Positive	11 (40.7)	16 (59.3)		
CVD History				
Pre-Heart Failure	30 (21.4)	110 (78.6)	17.4***	(3.7; 81)
Heart Failure	17 (81)	4 (19)		

*0.01 < p < 0.05, **p < 0.01 and ***p < 0.001.

**Table 6:** Multivariate logistic regression analysis for ARDS.

ARDS Model	Yes N (%)	No N (%)	OR	Bootstrap CI
Gender				
Male	21 (16)	107 (84)	2.316*	(1.073; 4.997)
Female	15 (31)	33 (69)		

*0.01 < p < 0.05, **p < 0.01 and ***p < 0.001.

**Table 7:** Multivariate logistic regression analysis for death.

Death Model	Yes Mean ± SD Or N (%)	No Mean ± SD Or N (%)	OR	Bootstrap CI
Age	71.9 ± 11.1	67.8 ± 12.5	1.019	(0.989; 1.05)
Gender				
Male	35 (27)	93 (73)	1.369	(0.651; 2.88)
Female	17 (35)	31 (65)		
Pulmonary history				
Negative	42 (28)	107 (72)	1.149	(0.434; 3.045)
Positive	10 (37)	17 (63)		
CVD history				
Pre-Heart Failure	41 (27)	113 (73)	3.27*	(1.163; 9.198)
Heart Failure	11(50)	11 (50)		

*0.01 < p < 0.05, **p < 0.01 and ***p < 0.001.

**Table 8:** Multivariate logistic regression analysis for sepsis.

Sepsis Model	Yes N (%)	No N (%)	OR	Bootstrap CI
CVD history				
Pre-Heart Failure	24 (16)	129 (84)	3.72**	(1.43; 9.67)
Heart Failure	9 (41)	13 (59)		

*0.01 < p < 0.05, **p < 0.01 and ***p < 0.001.

## 4 Discussion

This study focused on cardiac and inflammatory markers and how taking ACE_I_ and ARB affected their trending during COVID-19 infection. We found that patients taking ACE_I_ or ARB had less elevation in troponin T during admission. Troponin T could be elevated for many reasons, but in general increased stress on the heart may lead to an increase in troponin [12]. Moreover, patients taking ACE_I_ or ARB had lower peak levels of the inflammatory markers IL-6 and CRP.

This study did not show any statistically significant differences between patients taking ACE_I_ or ARB and the control group when we compared the proportions of ARDS, sepsis and death. As previously shown, peak troponin levels were more elevated in the control group, and the results showed that the ACE_I_ or ARB group had a lower odds ratio (0.419, p < 0.2) of having an elevated troponin on admission.

At the start of the pandemic there were some randomized controlled trials (RCTs) that investigated the effect of ACE_I_ and ARB during COVID-19 hospitalization. The ACE_I_-COVID trial investigated the risk of end organ failure in patients taking ACE_I_ or ARB. The study found that there was a higher risk of death 30 days after the infection and a higher risk of end organ damage in patients taking ACE_I_ and ARB [13]. The BRACE CORONA study looked at patients who are on chronic ACE_I_ and ARB treatment and found that there was no difference between patients taking these medications or other antihypertensives and the prognosis and risk of death after COVID infection [14]. The REPLACE COVID trial also found that there was no difference in the risk of death and other prognostic factors between patients taking ACE_I_ and ARB compared to patients taking other antihypertensives [15]. A recent meta-analysis reviewed 47 studies which investigated the effects of ACE_I_ and ARB on COVID-19 patients. The results were in favor of the hypothesis that ACE_I_ and ARB have protective effects in COVID-19 patients. The meta-analysis found that death and ICU admissions rates are lower in the study group [16].

The idea that discontinuation of ACE_I_ and ARB could lead to lower levels of ACE2 and thus less binding of the COVID-19 spike protein to the lungs and subsequently lower viral load in the body is not consistent with our results. If this were the case, we would have had lower levels of inflammatory markers in patients not taking ACE_I_ or ARB, which was not the case. But the higher levels of ACE2 in circulation, which is in part the natural response of the body to inhibition of the RAAS system by ACE_I_ and the ARB [6], could explain the observed lower levels of troponin.

Despite the fact that average values of CRP in blood on the day of admission were significantly lower in patients treated with ACE_I_/ARB compared to patients not taking these medications (Table 2), evidence for an anti-inflammatory effect of these medications, RAS inhibition had no effect on mortality of these patients. According to the work of Fang Liu and colleagues, COVID-19 patients with blood CRP values greater than 41.8 mg/L are the most likely to develop severe disease [17]. In addition, Guyi Wang and colleagues conclude that an optimal threshold value of 26.9 mg/L of CRP could be a valuable marker to anticipate the possibility of aggravation of adult patients with non-severe COVID-19 [18]. Thus, it is possible that the CRP values achieved in our study are high enough to determine a similar level of severity and prognosis in both groups. On the other hand, in a prospective clinical trial, Mariano Duarte and colleagues, using the ARB telmisartan in high doses of 160 mg/day vs. standard care in hospitalized patients with COVID-19 not in intensive care before 4 days from the onset of symptoms, report a significant decrease in plasma CRP values in the patients treated with the ARB on days 5 and 8 [19]. The CRP values on the day of admission, both in the patients in the treatment arm and in the control arm, were higher than the threshold values of greater risk of severity indicated above. Treatment with telmisartan caused a decrease in plasma CRP concentrations to values below said thresholds (day 5: 38.3 ± 50.8 mg/L, day 8: 23.7 ± 34.7 mg/L), while the values in the control group remained above said thresholds (day 5: 60.6 ± 69.5 mg/L, day 8: 63.0 ± 81.9 mg/L). In parallel, a marked decrease of 81% was observed in the mortality of patients in the group treated with telmisartan. Recently, these results of high-dose telmisartan in the treatment of patients with COVID-19 have been discussed from the clinical and pharmacological point of view [20,21].

## 5 Conclusion

This study supported available evidence that inhibition of the RAAS with ACE_I_ and 10.13039/100004800ARB can be continued safely for patients with COVID-19 infection. Although these drugs were not found to be beneficial for the prevention of ARDS, sepsis, or death, they proved to decrease the inflammatory markers in the body. Patients taking ACE_I_ and ARB showed lower levels of troponin, which correlates with less stress on the heart and the cardiovascular system. This finding needs to be further investigated by following up with patients by means of cardiac imaging to investigate the effect of COVID-19 infection on cardiac remodeling.

## Author contribution statement

Wissam Mekary: Conceived and designed the experiments; Performed the experiments; Analyzed and interpreted the data; Wrote the paper. Souha Fares, Farah Abdulhai, Mathias Mericskay: Conceived and designed the experiments; Analyzed and interpreted the data. Gaelle Massoud: Analyzed and interpreted the data. Marwan Refaat: Conceived and designed the experiments. George W. Booz: Analyzed and interpreted the data; Wrote the paper. Fouad A. Zouein: Conceived and designed the experiments; Analyzed and interpreted the data; Wrote the paper.

## Data availability statement

Data will be made available on request.

## Funding

This work was supported by grants from the 10.13039/100007688American University of Beirut 10.13039/100019603Faculty of Medicine [grant number 103944] and by 10.13039/501100004794Centre National de la Recherche Scientifique (CNRS) [grant number 104230] to FAZ. FAZ and M.M. are supported by the Agence nationale des recherches (ANR) et l’Agence française de développement (10.13039/501100011061AFD) [ANICOV-HF].

## Additional information

No additional information is available for this paper.

## Declaration of competing Interest

The authors declare that they have no known competing financial interests or personal relationships that could have appeared to influence the work reported in this paper.
